RETRACTED

# Inhibition of microRNA-299-5p sensitizes glioblastoma cells to temozolomide via the MAPK/ERK signaling pathway

**DOI:** 10.1042/BSR20181051

**Published:** 2018-09-12

**Authors:** Yujiang Peng, Xijun He, Huihui Chen, Hongyu Duan, Bo Shao, Fan Yang, Huiyong Li, Pengxiang Yang, Yu Zeng, Jinrong Zheng, Yongsheng Li, Jiachang Hu, Liguo Lin, Lingfang Teng

**Affiliations:** 1 Department of Neurosurgery, The First People’s Hospital of Wenling, Zhejiang Province 317500, China; 2 Department of Neurosurgery, Taizhou Cancer Hospital, Zhejiang Province 317500, China; 3 Department of Neurosurgery, The Hospital of Integrated Traditional Chinese and Western Medicine of Taizhou, Zhejiang Province 317523, China; 4 Department of Neurosurgery, The Dongfang Hospital of Wenling, Zhejiang Province 317525, China; 5 Department of Neurosurgery, Taizhou Orthopedics Hospital, Zhejiang Province 317500, China

**Keywords:** Glioblastoma (GBM), Golgi phosphoprotein 3 (GOLPH3), invasion, miR-299-5p, proliferation, temozolomide

## Abstract

Glioblastomas (GBMs) are a lethal class of brain cancer, with a median survival <15 months in spite of therapeutic advances. The poor prognosis of GBM is largely attributed to acquired chemotherapy resistance, and new strategies are urgently needed to target resistant glioma cells. Here we report a role for *miR-299-5p* in GBM. The level of *miR-299-5p* expression was detected in glioma specimens and cell lines by qRT-PCR. Luciferase reporter assays and Western blots were performed to verify GOLPH3 as a direct target of *miR-299-5p. In vitro* cell proliferation, invasion, cell cycle distribution, and apoptosis were assessed to determine whether or not *miR-299-5p* knockdown sensitized GBM cells to temozolomide (TMZ). We demonstrated that *miR-299-5p* levels were up-regulated in the GBM groups compared with the normal control group. The highest expression of *miR-129-5p* occurred in the highest GBM stage. *miR-299-5p* knockdown significantly inhibited the MAPK/extracellular signal-regulated kinase (ERK) signaling pathway. We also showed that *miR-299-5p* knockdown enhanced sensitivity of GBM cells to TMZ both *in vitro* and *in vivo* by inhibiting cell proliferation and invasion and promoting apoptosis. In addition, we demonstrated that GOLPH3 is a novel functional target of *miR-299-5p*. GOLPH3 regulates the MAPK/ERK axis under *miR-299-5p* regulation. In conclusion, we identified a link between miR-299-5p expression and the GOLPH3/MAPK/ERK axis, thus illustrating a novel role for *miR-299-5p* in GBM.

## Background

Glioblastoma (GBM) is the most common and destructive malignant brain tumor, accounting for approximately 30% of all the tumors in the central nervous system and 80% of malignant brain tumors [1–3]. Despite multimodality treatment, such as neuroimaging, surgery followed by phototherapy, radiotherapy, and adjuvant temozolomide (TMZ) chemotherapy, the prognosis of GBM patients is still unsatisfactory [4,5]. GBM is considered to be a primary brain tumor originating from glial stem or progenitor cells. Traditionally, GBM can be divided into astrocytomas, oligodendrocytomas, or ependymomas according to the histology, and divided into WHO grades I–IV according to the degree of malignancy [6,7].

RETRACTED

MiRNAs are small, non-coding RNA molecules (18–22 nts in length) that regulate target mRNAs by directly binding to mRNAs to degrade the mRNA or inhibit translation [8–10]. miRNAs can be used as tumor suppressors or oncogenes (oncomiRs) through negative regulation of the target mRNAs [11]. Previous studies have confirmed that miRNAs are involved in chemoresistance, most likely by regulating drug-resistant survival pathways [12,13]. A number of miRNAs have been identified to be involved in proliferation, invasion, and apoptosis of GBM [14,15]; however, no studies have focussed on the function of *miR-299-5p*. In the present study we determined the role of *miR-299-5p* in the MAPK signaling pathway. We hypothesized that *miR-299-5p* participates in the regulation of the MAPK pathway and affects the sensitivity of GBM to TMZ.

## Materials and methods

### Subjects

The study was approved by the Research Ethics Committee of The First People’s Hospital of Wenling. Each participant in the present study signed informed consent. Tissue specimens from patients with GBM and healthy brain tissue specimens were collected in the Department of Neurosurgery of The First People’s Hospital of Wenling. Tissue samples were collected from patients undergoing routine surgery between January 2011 and November 2016, including eight normal brain tissues, eleven WHO grade II, nine WHO grade III GBM tissues, and eight WHO grade IV GBM tissues. Brain tissue from healthy forensic cases (*n*=8) within the same age range as the examined glioma cases was collected. It served as a control in the gene studies. The clinical parameters of GBM patients were provided in Supplementary Table.

### Cell culture and chemical reagents

Human GBM cell lines (SNB19, LN308, T98G, A172, and U251) were purchased from the American Type Culture Collection (ATCC, Manassas, VA, U.S.A.). Normal astrocyte cells (NHAs) were purchased from Invitrogen (Carlsbad, CA, U.S.A.). Human GBM cell lines were cultured in Dulbecco’s modified Eagle’s medium (DMEM) with 10% inactivated FBS (Gibco-Life Technologies, Carlsbad, CA, U.S.A.), 100 U/ml of penicillin, and 100 mg/ml of streptomycin at 37°C in a humidified incubator with 5% CO_2_.

RETRACTED

### Lentivirus infection and gene transfection

Lentivirus containing *miR-299-5p* inhibitors (lv-*miR-299-5p*) or negative control (NC) was purchased from GenePharma (Shanghai, China). The human GBM cell lines, T98G and A172, were infected with a viral suspension. pcDNA3 or pcDNA3-GOLPH3 plasmids was transfected using Lipofectamine 2000 reagent (Invitrogen) according to the manufacturer’s instructions.

### qRT-PCR

After 48 h of infection or transfection, cells were collected for RNA and protein extraction. The total RNA was separated by TRIzol (Invitrogen, CA, U.S.A.). According to the manufacturer’s protocol, *miR-299-5p* was detected by qRT-PCR with a one-step RNA PCR kit (Takara, Otsu, Shiga, Japan). A PrimeScript RT kit (Takara Biotechnology Co., Ltd., Dalian, China) was used to reverse the total RNA by oligo dT primers. GAPDH was used as an internal reference. The primers used for qPCR were as follows: GOLPH3 (forward, 5′-AGTCGTTCTTGGTGCTAGGTA-3′ and reverse, 5′-CCCTTCGATGCGCTTACTGC-3′). The levels of target gene expression were quantitated on a 7900HT system using SYBR Premix DimerEraser (Biosciences,Pittsburgh, PA, USA), and the relative quantitative value was calculated by 2^−ΔΔ*C*^_t_.

### Vector construction

The GOLPH3 expression plasmid, pcDNA3-GOLPH3, was constructed and cells were treated with lv-*miR-299-5p* or GOLPH3 plasmids. Twenty-four hours after transfection, the cell lysates were prepared by dual luciferase lysate buffer (Promega, Agora, Fitchburg Center, Fitchburg, WI, U.S.A.). Luciferase activity was detected using a Mithras LB940 Microplate Reader (Berthold Technologies GmbH, Bad, Germany). The possible *miR-299-5p* binding site on GOLPH3 3′-UTR was inserted into the XbaI site of the pLKO.1-puro vector (Addgene, Cambridge, MA, U.S.A.). According to the instruction, Lipofectamine 2000 (Thermo Fisher Scientific, Inc., Waltham, MA, U.S.A.) was used to transfect the constructed vector into HEK293T cells.

### Protein extraction, Western blot, and immunoprecipitation

GBM cells were washed with PBS and lysed using cold RIPA buffer (Pierce, Brebieres, France) containing the protease inhibitor, PMSF (Sigma, St. Louis, MO, U.S.A.). Nuclear and cytoplasmic protein were isolated from the cultured GBM cells using a DUALXtract nuclear and cytoplasmic protein extraction kit (Dualsystems Biotech, Schlieren, Switzerland). The protein lysates were separated by SDS/PAGE and transferred on to PVDF membranes (Roche, Basel, Switzerland). The membranes were immunized with specific antibodies according to the standard experimental protocol. The antibody-labeled protein bands on the membrane were detected by G: BOX F3 (Syngene, Cambridge, U.K.). Cells were lysed by IP lysis buffer (Pierce, Rockford, IL, U.S.A.) in the immunoprecipitation assay. Membranes were incubated with the primary antibodies overnight at 4˚C. The following antibodies were used: rabbit anti-phosphorylated extracellular signal-regulated kinase (p-ERK; 1:1,000 dilution, catalog number NKC20314), GOLPH3 (SOX17; 1:1000 dilution, catalog number LUY13423), p-AKT (1:1000 dilution, catalog number ZYS01775), and GAPDH (1:1000 dilution, catalog number KC02335) (Sigma–Aldrich; Merck KGaA, Darmstadt, Germany). Membranes were subsequently incubated with a horseradish peroxidase-labeled goat anti-rabbit secondary antibody (1:5000 dilution; Beijing Solarbio Science and Technology, Co., Ltd., Beijing, China) at 37°C for 2 h.

RETRACTED

### Immunofluorescence analysis

Cells were infected with lv-*miR-299-5p* or NC for 48 h, and fixed in cold methanol for 2 min. Then, the cells were thrice-washed in PBS and incubated in blocked buffer for 30 min at room temperature. Next, cells were incubated with GSK3β and E2F1 (Abcam, Cambridge, MA, U.S.A.) at 4°C overnight after washing with PBS. Then, the cells were washed and incubated with the secondary antibody. The cells were stained by DAPI and observed under a fluorescence microscope (Thermo Fisher Scientific, Carlsbad, MA, U.S.A.) [16].

### Colony formation, invasion, cell cycle distribution, and apoptosis analysis

GBM cells (2000 cells/well) treated by lv-*miR-299-5p*, lv-NC, GOLPH3 plasmid, or nimotuzumab were placed in six-well plates containing fresh complete growth medium and the cells formed visible colonies. Cell colonies were fixed in cold methanol, then stained with 0.1% Crystal Violet for 15 min, photographed, and counted after washing and air drying. The cell invasion assay was performed using Corning Transwell insert chambers (Corning, New York City, NY, U.S.A.) and BD Matrigel invasion chambers (BD Biosciences, Bedford, MA, U.S.A.). The cells were added to the chamber and incubated for 24 h at 37°C. The cells in the lower chamber were fixed with 20% methanol and stained with 0.1% Crystal Violet, then photographed and counted.

### Detection of cell cycle by flow cytometry

The pre-treated T98G and A172 cells were fixed with 70% ethanol after washing with PBS and digested by trypsin. After washing, the cells were incubated in PBS containing propidium iodide and nuclease A (Sigma) at 37°C for 30 min. Cell cycle distribution was measured by DNA staining with DAPI dihydrochloride. Data of three independent experiments were expressed as the mean ± S.D. Forty-eight hours after transfection, the cells were collected, washed, and suspended in the dye buffer. An Annexin V-FITC apoptosis detection kit (KeyGEN Biotech, Nanjing, China) was used for analysis. The distribution of apoptosis in each sample was then determined by FACS. Annexin V-positive cells were considered as apoptotic cells.

RETRACTED

### Statistical analysis

GraphPad Prism software (GraphPad Software, Inc., San Diego, CA, U.S.A.) was used for statistical analysis. Statistical analysis included Student’s *t* test (two-tailed) and Pearson correlation analysis. A *P*<0.05 was regarded as statistically significant.

## Results

### Overexpression of *miR-299-5p* in GBM tissues

We first detected the expression of *miR-129-5p* in 28 GBM tissue samples and 8 normal brain tissue samples. Compared with the normal brain tissues, the expression of *miR-129-5p* in different GBM groups was up-regulated, while *miR-129-5p* in the WHO grade IV GBM group was the highest (Figure 1A and 1B). The expression of *miR-299-5p* was negatively correlated with the expression of *RASSF6* mRNA in tumor tissues by Spearman correlation analysis (Figure 1C). Then, we detected the expression of *miR-299-5p* in five GBM cell lines and NHA cells by qPCR. Compared with NHA, *miR-299-5p* was overexpressed in GBM cells (Figure 1D), indicating that *miR-299-5p* was up-regulated in GBM cells. In addition, qPCR showed that the expression of *miR-299-5p* in T98G and A172 cells was decreased by 78.6 and 76.3%, respectively, after transfection with lv-*miR-299-5p* (Figure 1E). Therefore, we chose these two cell lines for further functional analysis.

**Figure 1:** Overexpression of *miR-299-5p* in GBM tissue (**A**) The relative expression of *miR-299-5p* in 28 GBM tissue samples and 8 normal brain tissue samples. (**B**) Twenty-eight GBM tissues were divided into three groups: 11 WHO grade II tissues; 9 WHO grade III tissues; and 8 WHO grade IV tissues. The relative expression of *miR-299-5p* in normal brain tissue samples and GBM tissue samples was detected. *P*<0.0001 (**C**) Correlation between *miR-299-5p* and *GOLPH3* mRNA in 28 GBM tumor tissues was analyzed by Spearman correlation analysis (R^2^ = 0.4463, *P*<0.0001). (**D**) The expression of *miR-299-5p* in total RNA of GBM cell lines and NHA cells by qRT-PCR. Data are shown as the average fold of *miR-299-5p* expression in each GBM cell line compared with NHA. (**E**) The expression of *miR-299-5p* in GBM cells with or without lv-*miR-299-5p* infection detected by qPCR. *P<0.05, **P<0.01, ***P<0.001.

### Knockdown of *miR-299-5p* inhibited proliferation and invasion of GBM cells

We detected the effects of *miR-299-5p* knockdown on the proliferation and survival of T98G and A172GBM cells. Compared with lv-NC-treated cells, lv-*miR-299-5p* significantly inhibited colony forming ability (48.2 and 38.7%, respectively; Figure 2A). To detect the potential role of *miR-299-5p* in tumorigenesis, lv-*miR-299-5p* or lv-NC were infected into T98G cells. The luciferase bioluminescence imaging system showed that compared with the lv-NC group, knockdown of *miR-299-5p* in T98G cells significantly reduced the tumor (Figure 2B). These results indicated that *miR-299-5p* inhibited the tumorigenicity of GBM cells both *in vitro* and *in vivo*. Then, we examined how *miR-299-5p* affected the invasion and apoptosis of GBM cells. T98G and A172 cells were infected with lv-*miR-299-5p* for 48 h, and a significant increase in G_1_-phase arrest in these cells was noted (Figure 2C). Compared with lv-NC-treated cells, the invasiveness of lv-*miR-299-5p*-transfected cells were significantly reduced (Figure 2D). Apoptosis and the cell cycle of GBM cells transfected with lv-*miR-299-5p* (T98G and A172) were analyzed by flow cytometry, and we found that lv-*miR-299-5p*-transfected cells (T98G and A172) had a significant apoptosis rate (Figure 2E).

RETRACTED

**Figure 2:** Knockdown of *miR-299-5p* inhibited proliferation and invasion of GBM cells (**A**) T98G and A172GBM cells were treated with lv-NC or lv-*miR-299-5p*. (**B**) T98G cells pre-treated with luciferase reporter of lv-NC or lv-*miR-299-5p* were implanted into mice. The quality of tumor was detected by bioluminescence. **P<0.01 (**C**–**E**) T98G and A172 GBM cells were infected with NC or lv-*miR-299-5p*. The cell cycle distribution and apoptosis were detected after 48 h. After the cells were seeded in Transwell chambers for 24 h, cell invasion ability was analyzed. Three replicates per group, three independent experiments per group. *P<0.05.

### GOLPH3 is the direct target of *miR-299-5p*

Next, we used the 3′-UTR fragment of the GOLPH3 transcript (containing the *miR-299-5p* binding site) to analyze luciferase reporter (Figure 3A). Western blot analysis showed that the expression of GOLPH3 protein increased significantly in lv-*miR-299-5p*-infected GBM cells (Figure 3B). Compared with lv-NC infection, lv-*miR-299-5p* and WT GOLPH3 3′-UTR plasmid co-transfected T98G and A172 cells transiently, resulting in a significant increase in the activity of the luciferase reporter gene. GOLPH3 plasmid was successfully transfected into T98G and A172GBM cells (Figure 3C,D). GOLPH3 significantly inhibited proliferation and invasion of GBM cells (Figure 3E–G). GOLPH3 induced G_1_ phase arrest and increased apoptosis in GBM cells (Figure 3H).

**Figure 3:** GOLPH3 was the direct target of *miR-299-5p* (**A**) The 3′-UTR fragment of GOLPH3 containing predicted *miR-299-5p* target sites was fused downstream of luciferase gene. (**B**) The expression of GOLPH3 protein in T98G and A172 cells transfected with NC or lv-*miR-299-5p* was detected by Western blot analysis. (**C**) The human GOLPH3 3′-UTR luciferase reporter plasmid and NC or lv-*miR-299-5p* was co-transfected into T98G and A172GBM cells, as shown. Luciferase activity was detected after 48 h. (**D**) The expression of GOLPH3 protein was detected by Western blot after GOLPH3 expression or control plasmid was transfected into cells for 48 h. (**E**–**H**) Overexpression of GOLPH3 reversed the effect of *miR-299-5p* on GBM cell proliferation (E), cell cycle distribution (F), invasiveness (G), and apoptosis (H). *P<0.05. Three replicates per group, three independent experiments per group.

RETRACTED

### Synergistic effect of *miR-299-5p* inhibition and nimotuzumab on GBM cells and xenograft models

We further explored whether or not *miR-299-5p* inhibition had synergistic effect with nimotuzumab. T98G and A172 cells were treated with nimotuzumab (100 μg/ ml) for 24 h, then infected with lv-*miR-299-5p* or mimics control. After 4 days of lentivirus infection, cell proliferation, cell cycle distribution, invasiveness, and apoptosis were assessed. Lv-*miR-299-5p* enhanced the inhibitory effect of nimotuzumab on cell proliferation and invasion (Figure 4A,B). Flow cytometry analysis showed that more cells of the combination group were arrested in the G_1_ phase. In addition, cell apoptosis increased after combined treatment of nimotuzumab and lv-*miR-299-5p* (Figure 4C,D). Compared with nimotuzumab alone, combined treatment with nimotuzumab and lv-*miR-299-5p* significantly reduced tumorigenesis (Figure 4E). The results of Kaplan–Meier survival curve showed that combined treatment significantly prolonged the survival time (Figure 4F).

**Figure 4:** Lv-*miR-299-5p* enhanced the sensitivity of GBM cells to nimotuzumab in a mouse xenograft model (**A**–**D**) As shown, T98G and A172 cells were treated with nimotuzumab (100 μg/ml). After 24 h, the cells were infected with lv-*miR-299-5p* or no treatment. Cell proliferation, cell cycle distribution, invasion, and apoptosis in different groups were assessed. (**E**) Bioluminescence images of nude mice with implanted tumors and treated with nimotuzumab and/or lv-*miR-299-5p*. (**F**) The survival rate of mice was improved after combined treatment. *P<0.05 Three replicates per group, three independent experiments per group.

### *MiR-299-5p* regulates the responsiveness of GBM cells to TMZ via the GOLPH3-GSK3β-E2F1 pathway

Western blot analysis showed that *miR-299-5p* knockdown reduced the level of p-AKT and p-ERK in T98G and A172 cells (Figure 5). U0126 (MEK1/2 inhibitor) increased GOLPH3 expression in *miR-299-5p* knockdown T98G and A172 cells; however, the inhibitor of PI3K/AKT and LY294002 did not affect the expression of GOLPH3. These results suggested that *miR-299-5p* may induce malignant biological behaviors of GBM cells by activating the MAPK/ERK pathway and down-regulating GOLPH3.

RETRACTED

**Figure 5:** *MiR-299-5p* regulated GOLPH3 expression via the MAPK/ERK pathway The expression of GOLPH3 after MEK inhibitor (U0126) and PI3K inhibitor (LY294002) treatment was detected by Western blot.

## Discussion

MiRNA is a small, non-coding RNA which may be an oncogene or tumor suppressor by inhibiting the expression of target genes [17]. The MAPK signaling pathway can also be regulated by many miRNAs [18]. For example, *miR-431* is down-regulated in human GBM and directly inhibited MAPK expression by targetting 3′-UTR [19]. In addition, *miR-155* inhibited activation of the Akt pathway independent of the inhibition of MAPK [20]. *MiR-299-5p* is located in the DLK1-DIO3 genomic locus at chromosome 14q32.31. Ectopic expression of *miR-299-5p* has been demonstrated in various carcinomas, including colorectal cancer, leukemia, and breast cancer [21–23]. A comprehensive analysis of miRNA and mRNA showed that hsa-*miR-299-5p* binds to osteopontin (OPN) and promotes the proliferation and migration of tumor cells [24]. *MiR-299* is dysregulated in estrogen receptor (ER)-positive breast cancer [25]. *MiR-299-5p* has an opposing role in acute myeloid leukemia (AML) depending on whether or not cytogenetic *miR-299-5p* is down-regulated in patients with t(11q23)/MLL rearrangement and up-regulated in t(15;17) cytogenetic subtypes [22]. *MiR-299-5*p significantly induced cell growth and cell cycle progression effects in acute promyelocytic leukemia cells through the suppression of p21Cip1/Waf1 pathway [26]. In Alzheimer’s disease mouse model, the decreased levels of *miR-299-5p* were found both in primary neurones under conditions of starvation and in hippocampi of APPswe/PS1dE9 mice [27]. In the current study we first demonstrated that *miR-299-5p* is up-regulated in human GBM cells. Studies have shown that miRNAs can affect the response of ovarian, pancreatic, and bladder cancers, and GBM to chemotherapy [28]. Zhang et al. [27] found that *miR-299-5p* was up-regulated in the lung adenocarcinoma cell line, H3255, which contains MAPK mutations and is highly sensitive to AG1478. Inhibition of *miR-21* enhanced AG1478-induced apoptosis in these lung cancer cells, which were moderately sensitive to AG1478 [29].

Because *miR-299-5p* could regulate the MAPK signaling pathway, we wondered whether or not *miR-299-5p* can enhance the sensitivity and potential mechanism of GBM to nimotuzumab *in vitro* and *in vivo*. We identified GOLPH3 as the potential target of *miR-299-5p* and performed the 3′-UTR luciferase assay to determine whether or not *miR-299-5p* binds to the 3′-UTR of GOLPH3. The relative luciferase activity of the *GOLPH3* gene in lv-*miR-299-5p*-infected GBM cells was significantly higher than lv-NC-infected cells. The findings were confirmed by Western blot analysis. Our results showed that the expression of GOLPH3 protein was significantly up-regulated in lv-*miR-299-5p*-infected cells. These results demonstrated that GOLPH3 was the direct target of *miR-299-5p*. In addition, we confirmed that *miR-299-5p* regulated the formation of β-catenin/HIF-1α complex. Both β-catenin and HIF-1α are important MAPK-related transcription factors. Finally, the current study showed that the proliferation and invasion of GBM cells were attenuated after combination treatment of lv-*miR-299-5p* and nimotuzumab, and the proliferation and invasiveness decreased. The similar results were confirmed in nude mice treated with both lv-*miR-299-5p* and nimotuzumab.

RETRACTED

## Conclusion

In conclusion, the present study demonstrated for the first time that *miR-299-5p* expression in GBM cells was significantly increased. *MiR-299-5p* regulated the MAPK pathway by directly targetting GOLPH3. We identified the survival-related miRNA, *miR-299-5p*, as a regulatory factor affecting MAPK reactivity. Our research may be of great significance for the development of new therapies in patients with GBM.

## Supporting information

**Supplement Table:** Clinical parameters of glioma patients (n = 28)

## Abbreviations

GAPDH: glyceraldehyde-3-phosphate dehydrogenase
GBM: glioblastoma
GOLPH3: golgi phosphoprotein 3
GSK3β: glycogen synthase kinase-3β
HIF-1α: hypoxia inducible factor-1α
IP: immunoprecipitation
MAPK: mitogen-activated protein kinase
NC: negative control
NHA: normal astrocyte cell
p-AKT: phospho-Akt
p-ERK: extracellular signal-regulated kinase
PI3K: phosphoinositide 3-kinase
qRT-PCR: quantitative reverse transcription polymerase chain reaction
RIPA: radioimmunoprecipitation assay
TMZ: temozolomide
